The article "Cyclic GAN Model to Classify Breast Cancer Data for Pathological Healthcare Task" was retracted in 2024. Reasons: signs of a paper mill; suspected computer-generated content; unreliable results or conclusions; concerns about the data.

# Cyclic GAN Model to Classify Breast Cancer Data for Pathological Healthcare Task

**DOI:** 10.1155/2022/6336700

**Published:** 2022-07-21

**Authors:** Pooja Chopra, N. Junath, Sitesh Kumar Singh, Shakir Khan, R. Sugumar, Mithun Bhowmick

**Affiliations:** ^1^School of Computer Applications, Lovely Professional University, Phagwara, Punjab, India; ^2^University of Technology and Applied Science Ibri, Oman; ^3^Department of Civil Engineering, Wollega University, Nekemte, Oromia, Ethiopia; ^4^College of Computer and Information Sciences, Imam Mohammad Ibn Saud Islamic University (IMSIU), Riyadh, Saudi Arabia; ^5^Department of Computer Science and Engineering, Saveetha School of Engineering, Saveetha Institute of Medical and Technical Sciences, Chennai 601205, India; ^6^Bengal College of Pharmaceutical Sciences and Research, Durgapur, West Bengal, India

## Abstract

An algorithm framework based on CycleGAN and an upgraded dual-path network (DPN) is suggested to address the difficulties of uneven staining in pathological pictures and difficulty of discriminating benign from malignant cells. CycleGAN is used for color normalization in pathological pictures to tackle the problem of uneven staining. However, the resultant detection model is ineffective. By overlapping the images, the DPN uses the addition of small convolution, deconvolution, and attention mechanisms to enhance the model's ability to classify the texture features of pathological images on the BreaKHis dataset. The parameters that are taken into consideration for measuring the accuracy of the proposed model are false-positive rate, false-negative rate, recall, precision, and *F*1 score. Several experiments are carried out over the selected parameters, such as making comparisons between benign and malignant classification accuracy under different normalization methods, comparison of accuracy of image level and patient level using different CNN models, correlating the correctness of DPN68-A network with different deep learning models and other classification algorithms at all magnifications. The results thus obtained have proved that the proposed model DPN68-A network can effectively classify the benign and malignant breast cancer pathological images at various magnifications. The proposed model also is able to better assist the pathologists in diagnosing the patients by synthesizing the images of different magnifications in the clinical stage.

## 1. Introduction

The most definitive criterion for detecting breast disorders is a histological examination of breast tissue [1]. To aid pathologists in diagnosis, the traditional auxiliary diagnostics employ edge detection to segment cell nuclei [2]. Support vector machines [3], random forest [4], and other machine learning-based approaches employ artificially derived features for modelling and classification [5, 6]. The classification accuracy is low because pathological pictures typically have considerable differences [7], feature extraction relies on high professional expertise, and comprehensive feature extraction is challenging. Deep learning can overcome the limits of manual feature extraction and extract complicated nonlinear characteristics automatically, which has become increasingly popular in the categorization of diseased pictures [8]. In literature [9] on the BreaKHis dataset, the classification accuracy of the patient-level and image-level classifications was 90 percent and 85.6 percent, respectively, based on the AlexNet model paired with the maximum fusion approach for classification. Literature [10] used a single-task CNN model to train two CNN (convolutional neural network). Breast cancer can occur in two different categories [22–24], namely, benign [25] and malignant [26], and is a difficult task for pathologists to identify the type of cancer. Benign tumors are not cancerous, but on the other hand, malignant tumors are cancerous. A benign tumor [27] can be formed anywhere on or in the patient's body when cells multiply more than they should or they do not die when they should [30, 31]. Therefore, different machine learning techniques like logistic regression, naïve Bayes, and SVM [28, 29] and deep learning techniques like CNN, RNN, and neural networks [32, 33] are used in the field of healthcare for the detection purposes [34, 35]. Multitask CNN is utilized to predict malignant subtypes in breast cancer tumors, and the accuracy rates of binary and quaternary classification at the patient level are 83.25 percent and 82.13 percent, respectively. Literature [11] calculated that the average accuracy of binary classification at the patient level is 91 percent, according to GoogLeNet's fine-tuning learning process. Literature [12] introduced the msSE-ResNet (multiscale channel squeeze and excitation) multiscale channel recalibration model, which has 88.87 percent classification accuracy for benign and malignant tumors. Literature [13] created the BN-Inception (batch normalization-inception) model, which ignores magnification during training and achieves an accuracy rate of 87.79 percent on 40 diseased images. Literature [14] extracted characteristics using frequency domain information and classified them using long short-term memory (LSTM) and gated recurrent unit (GRU), with a classification accuracy of 93.01 percent. These findings show that deep learning-based approaches for pathological picture categorization are successful.

The article "Cyclic GAN Model to Classify Breast Cancer Data for Pathological Healthcare Task" was retracted in 2024. Reasons: signs of a paper mill; suspected computer-generated content; unreliable results or conclusions; concerns about the data.

Inconsistency in staining is a common concern with different batches of pathology pictures. The classification accuracy will be reduced if these samples are used to train the classification model. Pathological pictures include rich textural characteristics and little semantic information. To increase classification accuracy, additional medium- and low-level characteristics must be extracted. To address the aforementioned issues, this research provides an approach based on CycleGAN and an upgraded DPN, as well as a color normalizing technique based on CycleGAN, to mitigate the influence of dyeing issues on classification accuracy. The DPN is used to extract and classify features automatically. To increase the picture classification accuracy, we use improvement methods including tiny convolution, deconvolution layer, and attention mechanism, as well as a discriminating approach based on confidence rate and voting mechanism.

The next section of the paper discussed some of the related work, followed by the algorithm description used in the research. Later on, the experiments involved in the research have been analyzed and finally conclusion has been discussed.

## 2. Related Work

### 2.1. CycleGAN Structure

In image generation, the generative adversarial network (GAN) [15] is commonly utilized. A generator and a discriminator form the foundation of the system. The loss function is continuously optimized to generate actual data, which is extremely close to pseudodata, through the game between the generator and the discriminator. The CycleGAN presented in literature [16] is a ring network structure based on GAN that can realize style transfer between unpaired images and ensure that the generated image's color changes while remaining consistent with the source image. The specifics have not changed.

Two generators and two discriminators make up CycleGAN.  Figure 1 depicts the CycleGAN model structure. The generator is one of them, since it is used to create *Y* domain style images from the *X* domain, and the generator will create the *Y* domain image. Restore the image of the *X* domain [36]. The discriminator is used to make the image generated by the generator as close to the image of the *Y* domain style as possible, and the discriminator is used to make the image generated by the generator as close to the original image of the original *X* domain as possible so that when the image style is transferred, the features of the original image in the original *X* domain remain. Cycle consistency allows the CycleGAN to create more accurate and dependable pictures. The CNN classifier can also assist the producer in concentrating on lesion regions and obtaining prediction results. The differentiator and classification can help the generator perform accurate and dependable generating operations [37]. The advantage of cyclic GAN is that this model is faster than CNN as the model is more realistic in operation [38, 39]. Another benefit is that it does not require more preprocessing but suffers from time and space complexity like CNN and RNN [40]. The sigmoid loss function has been considered in the research. The loss function for the overall training of *L*_GAN_ (*F*, *D*_*X*_, *Y*, *X*) CycleGAN consists of the following 3 parts.

1. The loss of *X* domain GAN, where the discriminator is *D*_*X*_ and the generator is *F*
2. The loss of *Y* domain GAN, where the discriminator is *D*_*Y*_ and the generator is *G*
3. Reconstruction error: *L*_cyc_ = *L*_cyc_^*x*^ + *L*_cyc_^*y*^

The total loss of CycleGAN is

(1) $$\begin{array}{c} L\left(G,F,D_{X},D_{Y}\right)=L_{\text{GAN}}\left(G,D_{Y},X,Y\right)+L_{\text{GAN}}\left(F,D_{X},Y,X\right)+\lambda L_{\text{cyc}}\left(G,F\right). \end{array}$$

In the formula, *λ* is the weight coefficient.

(1) *L*_GAN_ (*G*, *D*_*Y*_, *X*, *Y*): input the original *X* domain slice “*a*” into the generator to generate slice *a*′ with *Y* domain color features, and the discriminator judges whether slice *a*′ belongs to the *Y* domain. The loss of the *X* domain GAN is
  (2) $$\begin{array}{c} L_{\text{GAN}}\left(G,D_{Y},X,Y\right)=E_{y\sim p\text{data}\left(y\right)}\left[\log_{2}D_{Y}\left(y\right)\right]+E_{x\sim p\text{data}\left(x\right)}\left[\log_{2}\left(1-D_{Y}\left(G\left(x\right)\right)\right)\right],\\ \underset{G}{\min}\underset{D_{Y}}{\max}L_{\text{GAN}}\left(G,D_{Y},X,Y\right). \end{array}$$
(2) *L*_GAN_ (*F*, *D*_*X*_, *Y*, *X*): the original *Y* domain slice *b* is input to the generator to generate slice *b*′ with *X* domain color features, and the discriminator judges whether slice *b*′ belongs to the *X* domain. The loss of the *Y* domain GAN for
  (3) $$\begin{array}{c} L_{\text{GAN}}\left(G,D_{X},X,Y\right)=E_{x\sim p\text{data}\left(x\right)}\left[\log_{2}D_{X}\left(x\right)\right]+E_{y\sim p\text{data}\left(y\right)}\left[\log_{2}\left(1-D_{X}\left(F\left(y\right)\right)\right)\right], \end{array}$$
  where *F* represents the generator from the *Y* domain to the *X* domain, *D*_*X*_ is the discriminator, and *F*(*y*) is the generated false sample in the *X* domain. The goal of the generator *F* is to minimize *L*_GAN_ (*F*, *D*_*X*_, *Y*, *X*), and the objective of discriminator *D*_*X*_ is to maximize it, so the objective function is
  (4) $$\begin{array}{c} \underset{F}{\min}\underset{D_{X}}{\max}L_{\text{GAN}}\left(F,D_{X},Y,X\right). \end{array}$$
(3) cyc (*G*; *F*): ideally, the original slice “*a*” of the *X* domain and the restored slice *a*^″^ of the *X* domain should be the same, but in fact, there is a difference between *a* and *a*^″^, and the difference between slice *a* and slice *a*^″^ is counted as *L*_cyc_^*xLxcy*^. In the original *Y* domain, the difference between slice *b* and restored slice *b*^″^ in the *Y* domain is calculated as *L*_cyc_^*y*^

The article "Cyclic GAN Model to Classify Breast Cancer Data for Pathological Healthcare Task" was retracted in 2024. Reasons: signs of a paper mill; suspected computer-generated content; unreliable results or conclusions; concerns about the data.

### 2.2. DPN68 Network Structure

DPN is a dual-path structure network based on ResNeXt and DenseNet [17]. It combines the advantages of ResNeXt and DenseNet and changes the output of each layer in addition to parallel so that each layer can directly obtain all previous. The output of the layer makes the model more fully utilize the features.

The DPN68 network structure is shown in Table 1. After a 3 × 3 convolution operation and then a 3 × 3 maximum pooling operation, it enters the block operation (the content of [*a*] in Table 1). Among them, ×3 means 3 cycles, the block of this parameter, *G*, refers to how many paths (i.e., the number of groups) are divided in a block of ResNeXt, and +16 represents the number of channels added each time in a block in DenseNet. The original DPN68 network goes through Conv3, Conv4, and Conv5, and softmax is used for multiclassification.

Figure 2 depicts the block structure of the DPN. The ResNeXt channel is on the top, and the DenseNet channel is on the bottom. Following the addition of the upper and lower channels, a 33% convolution and an 11% dimension transformation are performed. The output is separated, the upper path is combined with the upper path's original input, and the lower path is merged with the lower path's original input, generating a DPN block.

### 2.3. Attention Model

The study of human eyesight led to the discovery of the attention mechanism. Humans must choose certain portions to focus on to devote limited visual information processing resources to life. Attention may be applied to the input picture in neural networks. To increase the categorization accuracy of benign and malignant tumors, we partially assign different weights [18].  Figure 3 depicts the structure of the attention layer.

Adding attention layers is achieved through 3 operations named squeeze, excitation, and scale [19].

#### 2.3.1. Squeeze Operation

Squeeze operation achieves feature compression for each channel through global pooling operation. The number of channels *C* remains unchanged so that the original size of the feature map of *H* × *W* × *C* becomes 1 × 1 × *C*. The formula is as follows:

(5) $$\begin{array}{c} z_{C}=F_{\text{sq}}\left(u_{C}\right)=\frac{1}{H\times W}\overset{H}{\underset{i=1}{\sum }}\overset{W}{\underset{j=1}{\sum }}u_{C}\left(i,j\right). \end{array}$$

In the formula, *u*_*C*_(*i*, *j*) is the element of the *i*-th row and the *j*-th column of the two-dimensional matrix output by the deconvolution operation.

The article "Cyclic GAN Model to Classify Breast Cancer Data for Pathological Healthcare Task" was retracted in 2024. Reasons: signs of a paper mill; suspected computer-generated content; unreliable results or conclusions; concerns about the data.

#### 2.3.2. Excitation Operation

The excitation operation reduces the feature dimension to the original 1/*n* through the fully connected layer, and after the activation of the ReLu function layer, it is restored to the original number of channels *C* through the fully connected layer, and the sigmoid function is used to generate the normalization weights.

(6) $$\begin{array}{c} s_{C}=F_{\text{ex}}\left(z_{C},W_{1},W_{2}\right)=\sigma \left(W_{2}\delta \left(W_{1}z_{C}\right)\right). \end{array}$$

In the formula, 0 < *s*_*C*_ < 1.0; *σ* represents the sigmoid function; *δ* represents the ReLu function, and the output is positive; *W*_1_ and *W*_2_ are the weight matrices of the two fully connected layers, respectively.

#### 2.3.3. Scale Operation

The scale operation introduces an attention mechanism by weighting the normalized weight *s*_*C*_ to the features of each channel; that is, the channel input is multiplied by the weight coefficient and assigns different weights to the features of different dimensions. The weighting process formula is as follows:

(7) $$\begin{array}{c} F_{\text{scale}}\left(u_{C},s_{C}\right)=s_{C}u_{C}. \end{array}$$

## 3. Algorithm Description

To better enhance the pathological image classification accuracy, a model structure based on CycleGAN and DPN for image classification of pathological image is proposed, as shown in Figure 4.

The CycleGAN is used for color normalization of pathological images, that is, to convert pathological images of different colors to the same color to reduce the impact of color on classification. The DPN uses a 68-layer DPN model with an attention mechanism, which enhances the ability to classify pathological images.

1. Perform overlapping slice processing on the pathological images with the original size of 700 × 460 pixels in the BreaKHis dataset. Each original image is converted into 12 pathological image slices with the size of 224 × 224 pixels
2. According to the different colors of the pathological images in the dataset, a target color is selected, and the remaining color images are converted into target colors based on the CycleGAN to achieve color normalization
3. Data enhancement is carried out for the problem of unbalanced data. Data augmentation is carried out by flipping, rotating, fine-tuning, brightness, and contrast [20] so that the number of benign slices and the number of malignant slices reach a basic balance
4. Based on the DPN68 network, improve the classification accuracy by adding small convolution and deconvolution and introducing attention mechanism

The article "Cyclic GAN Model to Classify Breast Cancer Data for Pathological Healthcare Task" was retracted in 2024. Reasons: signs of a paper mill; suspected computer-generated content; unreliable results or conclusions; concerns about the data.

### 3.1. Color Normalization of Pathological Images Based on CycleGAN

Due to the different doses of different doctors when dyeing pathological images, it is easy to cause different shades of stained pathological images, especially pathological images of different periods, which are very different, such as original slice *a* and original slice *b* in Figure 5. The training and modeling of pathological images with different staining will lead to a decrease in the accuracy of the model, so it is necessary to perform color normalization on pathological images. The red arrows in Figure 5 indicate cycle loss, yellow arrows indicate GAN loss, and dotted arrows indicate *L*_cyc_.

The generators *G* and *F* in CycleGAN have the same structure, which consists of three parts: encoder, converter, and decoder. The structures of discriminator *D*_*X*_ and discriminator *D*_*Y*_ are the same, and they are composed of 5-layer convolutional neural networks.

The pathological image slices in the dataset are classified by color, and one of them is used as the *Y* domain image (target color image), and the rest of the color categories are used as the *X* domain image. The model framework of the pathological image color normalization based on CycleGAN is shown in Figure 5, the input is the *X* domain slice, and the output is the generated Y domain slice.

As shown in Figure 5, the input *X* domain slice *a* pass through the generator *G* to generate slice *a*′ with the *Y* domain coloring feature, and the generator *G* continuously competes with the discriminator *D*_*Y*_ to make the generated slice color as close to the *Y* domain as possible. Then input to the generator *F*, a restored slice *a*^″^ dyed in the *X* domain is generated. In theory, the restored slice and the original slice should be the same, and the error between them is *L*_cyc_. B m, y continuously optimized *L*_cyc_, the texture features during color conversion are guaranteed. The same is true from the *Y* domain to the *X* domain, as shown in the inner circle structure in Figure 5.

The trained CycleGAN model can color-normalize the input raw slices of different colors, while keeping the texture features unchanged. After color-normalizing all pathological image slices, the classification results can be prevented from being affected by factor effects of uneven dyeing.

### 3.2. Improved DPN68-A Pathological Image Classification Model

The proposed improved DPN68-A network structure is shown in Table 2. The improved network adds a 1 × 1 small convolution in the Conv1 layer and introduces a deconvolution layer and an attention layer in the original DPN-68 network.

The article "Cyclic GAN Model to Classify Breast Cancer Data for Pathological Healthcare Task" was retracted in 2024. Reasons: signs of a paper mill; suspected computer-generated content; unreliable results or conclusions; concerns about the data.

In the classification of pathological images, different from image classification tasks such as people, plants, and animals, it is necessary to extract high-level features for classification. Because the texture features of pathological images are more complex, it is more beneficial to use neural networks to extract the middle- and low-level features of pathological images. In the convolutional neural network, the size of the receptive field of a single node is affected by convolution kernel size in the feature map. The greater the convolution kernel, the more will be receptive field corresponding to a single node, the more abstract the extracted features, and the more difficult it is to focus on the image in the image. Detailed features: it is proposed to use a 1 × 1 small convolution in the Conv1 layer to transform the original image to obtain a new image; by connecting the ReLu activation function on the premise of keeping the size of the feature map (feature map) unchanged, the front the learning representation of one layer adds a nonlinear excitation, which allows the network to learn more complex nonlinear expressions, improves generalization ability, and reduces overfitting. Extracting more texture features from the original image enhances the expressive ability of the neural network.

Considering that the size of the feature map extracted from the input image after passing through the convolutional neural network is usually small, the deconvolution operation can enlarge the feature map, which helps the subsequent classifier to make a better judgment, so the deconvolution layer is added after Conv5.

Due to the different focus of distinguishing benign and malignant diseases in pathological images, it is necessary to assign different classification weights to different features and introduce an attention mechanism into the model. Through the three operations of squeeze, excitation, and scale in the attention layer, the normalization can be the weights are weighted to the features of each channel of the output of the deconvolution layer so that more classification weights are assigned to important features such as blood vessels, glands, and nuclei during classification, and less important features such as bubbles are assigned less classification weights.

### 3.3. Discrimination Strategy

When the image slice is used as the classification unit, a discriminative strategy combining confidence rate and majority vote is adopted. The classification results of multiple slices are integrated to obtain the final classification result of the image, which improves the classification accuracy of the pathological image in the network.

The article "Cyclic GAN Model to Classify Breast Cancer Data for Pathological Healthcare Task" was retracted in 2024. Reasons: signs of a paper mill; suspected computer-generated content; unreliable results or conclusions; concerns about the data.

For the *k* slices of each pathological image, let the number of slices classified as malignant be *k*_*nm*_, and the sum of confidence rates be CRM; the number of slices classified as benign is *k*_*nb*_, and the sum of confidence rates is CRB. The final classification result *T* is

(8) $$\begin{array}{c} T=\left\{\begin{array}{cc} 1, & k_{nb}>\frac{k}{2},\\ 0, & k_{nm}>\frac{k}{2}. \end{array}\right. \end{array}$$

The result that takes the majority of slices is the final result of the patient. If the number of benign slices in the classification result is equal to the number of malignant slices, the larger sum of confidence rates is taken as the final classification result of the image.

(9) $$\begin{array}{c} T=\left\{\begin{array}{cc} 1, & \text{CRB}>\text{CRM},\\ 0, & \text{CRM}>\text{CRB}. \end{array}\right. \end{array}$$

### 3.4. Algorithm Process

The proposed algorithm based on CycleGAN and improved DPN68-A network is as follows.

1. The original breast cancer pathological image (700 × 460 pixels) is processed by overlapping slices, and each pathological image corresponds to 12 pathological image slices with a size of 224 × 224 pixels
2. Pick out 2 pathological image slices of different colors in the pathological image slices, in which the *X* domain images are pathological image slices of different colors and the *Y* domain images are all pathological image slices of the target color
3. Train the CycleGAN model so that the model can output pathological image slices of different inputs as the same color. All data are color-normalized
4. Train and optimize the DPN68-A network
5. In the test phase, a fusion strategy combining majority voting and confidence rate is adopted, and the classification result of 12 slices corresponds to one image
6. Output the benign and malignant classification results of the image

## 4. Experimental Results and Analysis

### 4.1. Experimental Environment and Evaluation Indicators

#### 4.1.1. Experimental Environment

The following is a list of the hardware utilized in the experiment. The CPU is Intel Core i7-9750H@2.6 GHz; the memory is 16 GB; the operating system is 64-bit Windows10; the operating environment is Python 3.6; the GPU is NVIDIA GeForce GTX 1660Ti; and the hard drive capacity is 1 TB.

#### 4.1.2. Dataset and Data Processing

The breast cancer pathological image data collection BreaKHis was employed, which contains 7909 labelled breast cancer pathological pictures from 82 individuals with breast illness. 700 RGB three-channel pictures make up the data format. A total of 24 bits of color are used in the 460-pixel picture, with 8 bits in each channel.  Table 3 shows the particular distribution of pictures of benign and malignant tumors at various magnifications. The total number of images is divided by the number of cancerous images. Each picture is magnified five times: 50, 150, 250, and 500 times. The number of photos under 50x is 1986, 2048 for images under 150x, 2035 for images under 250x, and 1868 for images under 500x.

The article "Cyclic GAN Model to Classify Breast Cancer Data for Pathological Healthcare Task" was retracted in 2024. Reasons: signs of a paper mill; suspected computer-generated content; unreliable results or conclusions; concerns about the data.

Since the size of the input image required by the neural network is 224 × 224 pixels, the pathological image of breast cancer is sliced and segmented. Considering that many breast cancer pathological images contain a large number of bubbles, the image is displayed as white. If the nonoverlapping cutting method is used when classifying, it is easy to mistake such sliced images with a large proportion of white areas as normal images, reducing the accuracy of classification. Each image of 700 × 460 pixels is cut into 12 image slices of 224 × 224 pixels; as shown in Figure 6, by overlapping cutting, the same lesion area under different fields of view is repeatedly predicted to avoid false detection in the above situation.

In the BreaKHis dataset, the number of malignant patients and the number of malignant images are much higher than those of benign. The number of images is different for different patients, and the number of images between different disease categories varies greatly. To balance the data, 40x slice images are augmented. Augmentation methods include rotation, flipping, and fine-tuning contrast.

In the current research, there are usually two ways to establish datasets: dividing the dataset without isolating patients and dividing the dataset with isolated patients. The former does not consider patients and randomly divides the pathological image data into training set and test set, which will lead to pathological images of a certain patient may exist in both the training set and the test set. The model classification accuracy of this type of method is usually high, but its application value in specific clinical settings is limited. The latter isolates patients when dividing to ensure training data and testing data. The data is completely independent at the patient level, and the classification model established in this way has better practical application. Isolate patients and divide them into threefold.  Table 4 shows the specific distribution of benign and malignant sections.

#### 4.1.3. Evaluation Criteria

The classification performance of the model was evaluated from two aspects: patient level and image level.

*(1) Image-Level Accuracy*.

(10) $$\begin{array}{c} I=\frac{N_{r}}{N_{\text{all}}}, \end{array}$$

where *N*_all_ is the number of pathological images in the validation set and test set and *N*_*r*_ is the number of images that is correctly classified.

The article "Cyclic GAN Model to Classify Breast Cancer Data for Pathological Healthcare Task" was retracted in 2024. Reasons: signs of a paper mill; suspected computer-generated content; unreliable results or conclusions; concerns about the data.

The false detection rate is also known as type I error which is the probability that a false alarm will be raised; that is, the positive result will be given when the true value is negative.

(11) $$\begin{array}{c} \text{FPR}=\frac{\text{FP}}{\text{FP}+\text{TN}}=\frac{\text{FP}}{N_{b}}. \end{array}$$

The missed detection rate is also known as type II error which is the probability that a true positive will be missed by the test.

(12) $$\begin{array}{c} \text{FNR}=\frac{\text{FN}}{\text{TP}+\text{FN}}=\frac{\text{FN}}{N_{m}}. \end{array}$$

Recall rate:

(13) $$\begin{array}{c} \text{Recall}=\frac{\text{TP}}{\text{TP}+\text{FN}}=\frac{\text{TP}}{N_{m}}. \end{array}$$

The accuracy is

(14) $$\begin{array}{c} \text{Precision}=\frac{\text{TP}}{\text{TP}+\text{FP}}. \end{array}$$

*F*1 score is

(15) $$\begin{array}{c} F1\text{ score}=\frac{2\times \text{Precision}\times \text{Recall}}{\text{Precision}+\text{Recall}}. \end{array}$$

*(2) Patient-Level Accuracy*.

(16) $$\begin{array}{c} R=\frac{\sum P_{s}}{N_{p}}. \end{array}$$

In the formula, *P*_*s*_ is the classification accuracy rate of each patient, *P*_*s*_ = *N*_*rp*_/*N*_*np*_, where *N*_*np*_ is the number of pathological images of each patient and *N*_*rp*_ is the number of correctly classified images of each patient; ∑*P*_*s*_ is the classification accuracy of all patients is the sum of the rates; *N*_*p*_ is the total number of patients.

### 4.2. Experiment and Result Analysis

#### 4.2.1. Experiment 1: Color Normalization Comparison Experiment

This experiment compares the impacts of two distinct color normalizing techniques and is used to verify the usefulness of the suggested color normalization approach. In the color normalization comparison experiment, 300 benign and 300 malignant photos from the pathological image 40 dataset were chosen at random as the experimental data. The training and test sets were built in a 7 : 3 ratio, with no crossover between the patient samples in the training and test sets. We examined the effects of color normalization without color normalization, color normalization with the Vahadane technique [21], and color normalization with the CycleGAN model on detection accuracy via tests. For parameter fine-tuning, the detection model uses DPN68-A, which was introduced in this publication and is based on ImageNet-5K pretraining. For 100 iterations, the pretraining parameter transfer learning is applied, and the final accuracy is computed as the evaluation index.  Table 5 shows the outcomes of the experiment.

The article "Cyclic GAN Model to Classify Breast Cancer Data for Pathological Healthcare Task" was retracted in 2024. Reasons: signs of a paper mill; suspected computer-generated content; unreliable results or conclusions; concerns about the data.

The experimental results show that after the pathological images are color normalized, the classification accuracy improves significantly, indicating that uneven color affects the deep learning model for pathological image classification, because normalization eliminates the interference of different colors on the classification results. The CycleGAN model's data classification accuracy rate is 10% higher than without the normalization approach, and the false detection rate is 14.4 percent lower, the missed detection rate is 5.6 percent lower, and the accuracy rate is increased. The classification accuracy is increased by 2.22 percent, the false detection rate is lowered by 3.3 percent, the missed detection rate is reduced by 1.1 percent, and the accuracy is improved by 2.22 percent when compared to the Vahadane technique. It is clear that the color normalization strategy for the pathological pictures described in this study, based on CycleGAN, is successful.

#### 4.2.2. Experiment 2: Comparison of Different CNN Models

To verify the effectiveness of different CNN models, GoogLeNet, VGG16, ResNet34, ResNet101, and AlexNet were compared. The experiment was carried out based on Data1, Data2, and Data3, and the results are as follows and shown in Table 6.

It can be analyzed from the experimental results that the ResNet34 and ResNet101 models based on residual structure have significantly higher classification accuracy than GG16, AlexNet, and GoogLeNet at both the image level and the patient level. Among them, the best performing ResNet34 network is accurate at the image level compared with VGG16, the rate is improved by 5.42%, the false detection rate is reduced by 16.98%, the missed detection rate is reduced by 0.18%, and the patient-level classification accuracy rate is improved by 8.21%. Compared with the ResNet101 network with deeper network layers, the image-level classification accuracy rate increases 0.6% and 1.71% increase in the patient-level classification accuracy. The residual structure is more suitable for the classification of pathological images, but the more layers of the network, the better the performance is not necessary.

#### 4.2.3. Experiment 3: DPN68 Network Improvement Ablation Experiment

This experiment is used to verify the effectiveness of the proposed DPN68-A model. The experiment adopts the form of ablation experiment, comparing the original DPN68 network and DPN68 network adding small convolution and DPN68 adding results of small convolution, deconvolution, and attention layers. The experiments are carried out based on Data1, Data2, and Data3, and the results are shown in Table 7 and Figure 7. In Table 7, AUC is the area under the ROC curve.

The article "Cyclic GAN Model to Classify Breast Cancer Data for Pathological Healthcare Task" was retracted in 2024. Reasons: signs of a paper mill; suspected computer-generated content; unreliable results or conclusions; concerns about the data.

It can be seen from the experimental results that, compared with the original DPN68 network, the DPN68 network with a small convolutional layer has an increase of 0.96% in patient-level classification accuracy, 0.95% in image-level classification accuracy, 1.9% in false detection rate, and 1.9% in missed detection. Compared with the DPN68 network, the improved DPN68-A model has a 1.92% improvement in patient-level classification accuracy and a 2.2% improvement in image-level classification rate, the false detection rate is reduced 5.26%, and the missed detection rate is reduced by 0.5%. It can be seen that the improved model has greatly improved the classification accuracy at both the patient level and the image level, effectively improving the performance of the classification model. The ROC curve is shown in Figure 8. The AUC metric of the improved DPN68-A model is 1.36% higher than that of the DPN.

#### 4.2.4. Experiment 4: Comparison Experiment of DPN68-A Model with Different Deep Learning Methods

Single-task CNN method [10], improved deep convolutional neural network model [11], multiscale recalibration model [12], BN-Inception classification model [13], and the LSTM+GRU classification model [14] for comparison and the accuracy results at the patient level are shown in Figure 9.

The detection accuracy of the approach in this study is superior to other machine learning and deep learning methods at the patient level, as shown by the comparative findings. There is a 3.68 percent improvement, a 5.81 percent increase, a 6.89 percent improvement, and a 1.67 percent improvement over the Ming algorithm, Zhou method, and LSTM+GRU algorithm.

#### 4.2.5. Experiment 5: Test Experiments of DPN68-A at All Magnifications

To prove that the proposed DPN68-A model is also applicable at other magnifications, the ×100, ×200, and ×400 data were color-normalized, respectively. The model is trained and the classification accuracy is tested. The experimental results are shown in Table 8 and Figure 10.

According to the experimental results, it can be seen that DPN68-A has a good detection effect on pathological images of various magnifications and can better assist pathologists in diagnosing patients by synthesizing images of different magnifications in the clinical stage.

## 5. Conclusion

Aiming at the problem of high-precision detection of breast cancer pathological images, this paper proposes a color normalization method for pathological image slices based on CycleGAN, which reduces the influence of uneven staining on the classification of pathological images. It is proposed to use DPN to establish a detection model. A 1 × 1 small convolution is added to the network structure to enhance the nonlinear expression ability of the network and better capture the texture features of pathological images. By adding a deconvolution layer and an attention mechanism, the model can better allocate the intermediate features. The weight of the network improves the classification accuracy of breast pathological images. A discriminant strategy combining confidence rate and voting mechanism is proposed to improve the classification accuracy of patient-level lesions. Experiments show that the proposed DPN68-A network can classify benign and malignant breast pathological images. It has a good effect and has certain clinical application value. In the future, the segmentation network will be combined to accurately label malignant areas on the basis of correctly classifying malignant images, to achieve more accurate clinical auxiliary judgments.

The article "Cyclic GAN Model to Classify Breast Cancer Data for Pathological Healthcare Task" was retracted in 2024. Reasons: signs of a paper mill; suspected computer-generated content; unreliable results or conclusions; concerns about the data.

## Figures and Tables

**Figure 1:** CycleGAN structure.

**Figure 2:** Block structure of DPN.

**Figure 3:** Attention mechanism structure.

**Figure 4:** CycleGAN and DPN model.

**Figure 5:** CycleGAN pathological image color normalization model.

**Figure 6:** Overlapping cutting of pathological images.

**Figure 7:** Accuracy comparison of improved classification using DPN68 network.

**Figure 8:** ROC curves of network.

**Figure 9:** Comparison results of DPN68-A and other classification algorithms.

**Figure 10:** Comparison results of DPN68.

**Table 1:** DPN68 network structure.

Layer	DPN68 network structure
Conv1	3 × 3, 10, stride 2
	3 × 3 max pool, stride 2
Conv2	$\left[\begin{array}{cc} 1\times 1, & 128\\ 3\times 3, & 128,G=32\\ 1\times 1, & 256\left(+16\right) \end{array}\right]\times 3$
Conv3	$\left[\begin{array}{cc} 1\times 1, & 256\\ 3\times 3, & 256,G=32\\ 1\times 1, & 512\left(+32\right) \end{array}\right]\times 4$
Conv4	$\left[\begin{array}{cc} 1\times 1, & 512\\ 3\times 3, & 512,G=32\\ 1\times 1, & 1024\left(+32\right) \end{array}\right]\times 12$
Conv5	$\left[\begin{array}{cc} 1\times 1, & 1024\\ 3\times 3, & 1024,G=32\\ 1\times 1, & 2048\left(+32\right) \end{array}\right]\times 3$
	Global average pooling layer, 1000-dimensional fully connected layer, softmax classifier

**Table 2:** DPN68-A network structure.

Layer	DPN68 network structure
Conv1	1 × 1, 10, stride 1 3 × 3, 10, stride 2
Conv2~Conv5	Same as DPN68
Deconvolution layer	Deconv
Attenuation layer	Global pooling, fc, ReLu, fc, sigmoid, scale

**Table 3:** Number of benign and malignant tumor images with different magnifications.

*A*	*N*_*ib*_	*N*_*im*_	*N*_*i*_
50	645	1365	1986
150	654	1498	2048
250	687	1354	2035
500	535	1289	1868

**Table 4:** Benign and malignant section distribution.

*A*	*N*_*ib*_	*N*_*im*_	*N*_*i*_
Data1	23564	22789	46218
Data2	16658	22351	38451
Data3	17894	20846	38165

The article "Cyclic GAN Model to Classify Breast Cancer Data for Pathological Healthcare Task" was retracted in 2024. Reasons: signs of a paper mill; suspected computer-generated content; unreliable results or conclusions; concerns about the data.

**Table 5:** Benign and malignant classification comparison.

Method	FPR	FNR	Recall	Precision	*F*1 score	*I*
No normalization	23.9	9.2	91.21	79.12	84.35	84.22
Normalization by Vahadane's method	14.5	5.3	96.14	88.64	92.41	92.38
CycleGAN normalization	11.7	4.6	95.37	89.83	93.71	93.16

**Table 6:** Accuracy comparison of different CNN models.

Model	FPR	FNR	Recall	Precision
VGG16	37.11	8.19	80.25	83.01
AlexNet	30.59	12.60	83.49	85.81
GoogLeNet	31.78	11.04	84.71	84.48
ResNet34	20.98	8.97	88.91	91.41
ResNet101	21.81	9.10	87.46	88.94

**Table 7:** Accuracy comparison of improved classification using DPN68 network.

The Internet	FPR	FNR	Recall	Precision	*F*1 score	*I*	*R*	AUC
DPN68	13.84	7.1	94.12	95.15	94.02	92.15	91.94	94.12
DPN68+small convolution	9.98	6.8	92.94	93.64	93.87	91.94	92.48	93.96
DPN68-A	8.10	5.9	93.45	95.89	95.64	93.18	93.74	95.03

**Table 8:** DPN68-A results at all magnifications.

*A*	FPR%	FNR%	Recall%	Precision%	*F*1 score%	*I*%	*R*%
50	8.10	7.15	94.41	97.87	95.74	94.11	95.11
150	7.05	5.65	95.01	98.61	97.21	93.94	95.31
250	8.16	3.45	94.89	95.94	96.48	94.12	95.17
500	7.95	5.59	93.47	98.10	95.32	95.01	94.67

## Data Availability

The data shall be made available on request.
